# The Association of HMGB1 Gene with the Prognosis of HCC

**DOI:** 10.1371/journal.pone.0089097

**Published:** 2014-02-19

**Authors:** Jianbiao Xiao, Yi Ding, Jing Huang, Qisheng Li, Ying Liu, Wen Ni, Yuqin Zhang, Yanfei Zhu, Longhua Chen, Bin Chen

**Affiliations:** 1 Department of Radiation Oncology, Nanfang Hospital, Southern Medical University, Guangzhou, Guangdong, China; 2 Department of Science and Training, General Hospital of Guangzhou Military Command of People's Liberation Army, Guangzhou, Guangdong, China; 3 Department of Cancer Center, Affiliated Hospital of Guangdong Medical College, Zhanjiang, Guangdong, China; Icahn School of Medicine at Mount Sinai, United States of America

## Abstract

High-mobility group box 1 protein (HMGB1) is an evolutionarily ancient and critical regulator of cell death and survival. HMGB1 is a chromatin-associated nuclear protein molecule that triggers extracellular damage. The expression of HMGB1 has been reported in many types of cancers, but the role of HMGB1 in hepato cellular carcinoma (HCC) is unknown.The aim of this study was to analyze the roles of HMGB1 in HCC progression using HCC clinical samples. We also investigated the clinical outcomes of HCC samples with a special focus on HMBG1 expression. In an immunohistochemical study conducted on 208 cases of HCC, HMGB1 had high expression in 134 cases(64.4%).The HMGB1 expression level did not correlate with any clinicopathological parameters, except alpha fetoprotein (AFP) (*p* = 0.041) and CLIP stage (*p* = 0.007). However, survival analysis showed that the group with HMBG1 overexpression had a significantly shorter overall survival time than the group with a down-regulatedexpression of HMBG1 (HR = 0.568, CI (0.398, 0.811), *p* = 0.002). Multivariate analysis showed that HMGB1 expression was a significant and independent prognostic parameter (HR = 0.562, CI (0.388, 0.815), *p* = 0.002) for HCC patients. The ability of proliferation, migration and invasion of HCC cells was suppressed with the disruption of endogenous HMGB1 using small interfering RNAs. On the other hand, the ability of proliferation, migration and invasion of HCC cells was strengthened when the expression endogenous HMGB1 was enhanced using HMGB1 DNA. HMGB1 expression may be a novel and independent predictor for the prognosis of HCC patients. The overexpression of HMGB1 in HCC could be a novel, effective, and supplementary biomarker for HCC, since it plays a vital role in the progression of HCC.

## Introduction

Hepatocellular carcinoma (HCC) is a highly lethal cancer as its prognosis is typically poor in most patients. HCC is a lethal cancer, as it is the third leading cause of cancer deaths in East Asia and sub-Saharan Africa [1], [2]. In China, it is far more lethal given the fact that it is the second leading cause of cancer deaths in Chinese men [3]. In recent times, its incidence is also increasing steadily in the United States and Europe [4], [5]. HCC is generally with poor prognosis, given the fact thatthe 5-year survival rate is as low as 25–39% after surgery in patients [6]. In most cases, HCC (>80%) is diagnosedat an advanced stage. Chemotherapy and radiotherapy have limited efficacy in dealing with patients diagnosed with HCC at an advanced stage [7]. In case of HCC patients who have undergone of tumor resection, the recurrence rate can be as high as 50% in 2 years [8], [9]. Research studies have concluded that the poor prognosis of HCC is associated with several clinicopathological parameters, such as poorly differentiated phenotype, portal venous invasion and intrahepatic metastasis. However, the underlying mechanisms associated the development of HCC have not been understood completely.

HMGB1 was originally described as a nuclear non-histone DNA-binding protein that functions as a structural co-factor critical for proper transcriptional regulation in somatic cells [10]–[13]. HMGB1 is highly conserved through evolution [14], [15], and although it is produced by nearly all cell types, its nuclear localization can vary with development and age [13], [14]. Structurally, HMGB1 has 215 residues organized into two DNA-binding domains (named A-box and B-box), and a negative charged C-terminus. The two DNA-binding domains are similar in conformation despite to their limited amino acid identity [15], [16]. HMGB1 is a versatile protein with intranuclear and extracellular functions. HMGB1 is a highly conserved nuclear protein, because itacts as a chromatin-binding factor that bends DNA. HMGB1 alsoinstigates access to transcriptional protein assemblies located on specific DNA targets [17], [18]. HMGB1 acts as an extracellular signaling molecule during several cellular processes, such as inflammation, cell differentiation, cell migration, and tumor metastasis [19], [20]. Previous research studies have confirmed that HMGB1 is closely related with tumorigenesis, metastasis, and angiogenesis in a variety of malignancies, such as breast cancer [21], melanoma [22], gastric cancer [23], and colorectal cancer [24].An overexpression of HMGB1 occurs due to two main reasons: KIT mutation and genes instigating tumour growth and invasion [25]. Furthermore, HMGB1 overexpression has been associated with several undesirable activities: inhibition ofcaspase activation, increase in NF-*k*B activity, and up-regulation of c-IAP2.Thus, the overexpression of HMGB1 inhibits the apoptosis of cancer cells [24]. In this study, we investigated the expression of HMGB1 in primary HCC using immunohistochemical analysis. We also identifiedhow HCC was related with different kinds of clinicopathological features.Furthermore, we evaluatedthe prognostic significance of HMGB1expression in the survival of HCC patients.

## Materials and Methods

### Patients and tissue samples

The ethical approval of the use of these clinical materials for research purpose in this article, the association of HMGB1 gene with the prognosis of HCC, was given by the medical ethics committee of General Hospital of Guangzhou Military Command of People's Liberation(PLA). Participants allowed us to make research with their specimens and clinicopathologic data. Not until got their consent can we made follow –up with them. Verbal informed consents were provided by participants at first in this study, because telephone was the main way to get touch with participants. When they came back hospital to review their bodies, we had done written consents with them.And the ethics committee approved this consent procedure.

In this study, we investigated 208 patients, who were dignosed with primary HCC. The inclusion and exclusion criteria :(a)distinctive pathologic diagnosis,(b) without pre-operative anti-cancer treatment and distant metastases, (c) surgerical liver resection, (d) with a complete clinico-pathologic and follow-up data [26]. In the period extending from 1999 to 2002, we investigated these patients who had undergone conventional surgery at General Hospital of Guangzhou Military Command of PLA, Guangzhou City, Guangdong Province, China. Before surgery, these patients were not subjected to radiotherapy or chemotherapy. After completion of surgical procedure, they were followed up for 5 years, and their complete clinical data were collected. All primary HCC samples were taken from these 208 patients. These primary samples were fixed in 10% formalin and subsequently embedded in paraffin.Thereafter, they were sectioned consecutively at 4 µm stained by hematoxylin and eosin. According to the criteria of the World Health Organization (WHO) classification system, the histological types were independently assigned by twodouble-blinded pathologists.

### Cell lines preparation

The human hepatoma cell line HepG2, HCCLM6, Huh7, 97H, 97L, HCCLM3, BEL-7404 and a normal hepatocyte line (L02) were purchased from the cell bank of Chinese Academy of Sciences. These cell lineswere cultured in DMEM (Invitrogen, Carlsbad, USA) medium, which was supplemented with 10% fetal bovine serum (Invitrogen).All the cells were maintained at 37°C in a humidified atmosphere containing 5% CO_2_.

### Immunohistochemistry (IHC)

IHC staining was performed using a Dako Envision System (Dako, Denmark) in accordance with the manufacturer's recommended protocol. In this case, all paraffin sectionswere baked for 2 h at 65°C. These sections were 4 µm in thickness. Sections were first deparaffinized with xylene; then they were rehydrated with graded ethanol and distilled water. Thereafter, sections were submerged in EDTA antigenic retrieval buffer (pH 8.0) and subjected to microwave treatment. At this stage, these sections were treated with 0.3% H_2_O_2_ for 15 min to block the endogenous peroxidase.Now, the sections were treated with 5% normal goat serum for 30 min.Then, rabbit monoclonal anti-HMGB1 antibody (1∶150) (epitomics,USA) was incubated overnight with the sections at 4°C. After washing, the sections were incubated with HRP at 4°C for 30 min. For performing colour reactions, diaminobenzidine (DAB) was used. For negative controls, the antibody was replaced with normal goat serum.

### Semiquantitative analysis

The immunohistochemically stained tissue sections were scored separately by two pathologists, who were blinded according to specific clinical parameters. While conducting HMGB1 assessment, the entire tissue section was scanned and the scores were assigned accordingly. The staining intensity was scored as 0 (negative), 1 (weak), 2 (medium), and 3 (strong). The extentof staining was scored as 0 (0%), 1 (1–25%), 2(26–50%), 3 (51–75%), and 4 (76–100%). The scoring was done by taking into account the percentages of the positive staining areas in relation to the entire carcinoma-involved area or the entire section for the normal samples. The sum of the intensity and extent scores was used as the final staining score (0–7) for HMGB1. While performing statistical evaluation, tumours with a final staining score of ≥3 were considered as high HMGB1 expression. Final staining score between 1 to 3 were considered as low HMGB1 expression [27].

### Real-time quantitative RT-PCR (qRT-PCR)

Total RNA was extracted using Trizol reagent (takara, China) and reversed transcribed. Quantitative real-time PCR analysis was performed using ABI PRISM 7500 Real-Time PCR System (Applied Biosystems,USA). Each well (20 µl reaction volume) contained 10 µl Power SYBR Green PCR master mix (Applied Biosystems), 1 µl of each primer, and 1 µl template.The following primers were used:

HMGB1 5′-TAAGAAGCCGAGAGGCAAAA-3′

5′-AGGCCAGGATGTTCTCCTTT-3′,

β-actin 5′-AAGACGTACTCAGGCCATGTCC-3′

5′-GACCCAAATGTCGCAGTCAG-3′.

### Western blotting analysis

Cells were washed twice with cold phosphate-buffered saline(PBS) and lysed on ice with RIPA buffer (13 PBS, 1% NP40, 0.1% sodium dodecyl sulfate (SDS), 5 mM EDTA, 0.5% sodium deoxycholate and 1 mM sodium orthovanadate) containing protease inhibitors.

Protein lysates were resolved with 10% SDS polyacrylamide gel; then they were electro-transferred to polyvinylidene fluoride membranes (Immobilon P; Millipore, Bedford, MA) and blocked in 5% non-fat dry milk in Tris-buffered saline, pH 7.5 (100 mMNaCl, 50 mMTris and 0.1% Tween-20). Membranes were immunoblottedovernight at 4°C with anti-HMGB1 monoclonal antibody (epitomics) and anti-b-actin antibody (PROTEINTECH GROUP).Thereafter, the immunoblotted membranes were treatedwith their respective horseradish peroxidase-conjugated secondary antibodies. Signals were detected through enhanced chemiluminescence (Millipore, 2×250 ml).

### HMGB1 siRNA transfection

Cells were seeded onto a six-well plate for 24 h before transfection. In each well, 60 pmol of HMGB1 siRNA, S1(5′-CCCGUUAUGAAAGAGAAAUTT-3′), S2(5′-GCAGCUUAUACGAAAUAAUTT-3′) and scramble siRNA sequences (5′-UUCUCCGAACGUGUCACGUTT-3′) (Genepharma, Shanghai, China), and 4 µl of TurboFectsiRNA Transfection Reagentwere(Thermo Scientific, Lithuania)were added to Opti-MEM and mixed gently. The plate was incubated for 48 h until it was ready for further assay.

### HMGB1 DNA transfection

**HMGB1 DNA** is cDNA clone, which was purchased from GeneChem company in Shanghai, China. Cells were seeded onto a six-well plate for 24 h before transfection. In each well, 4 µg of human HMGB1 DNA or 4 µg of vector GV142(GeneChem, Shanghai, China), and 6 ul of TurboFect Transfection Reagent(Thermo Scientific, Lithuania) were added to serum-free DMEM and mixed gently. The plate was incubated for 48 h before being subjected for further assay.

### Cell Proliferation Assay

Cell suspension (100 ul/well) were Inoculated in a 96-well plate. The plate was pre-incubate in an incubator (humidified atmosphere; at 37°C, 5% CO2). 10 ul of the cell counting kit-8 (CCK-8) (Dojindo, Jap) solution were added to each well of the plate. The plate was incubated for 1–4 hours in the incubator. the absorbance of each well was measured at 450 nm using a microplate reader. All experiments were performed in triplicate.

### Tumour cell migration assay

Migration assays were performed using the cell chamber (BD, USA) according to the manufacturer's protocol. In this case, warm serum-free medium was added to the top of the cell chamber. Tumor cells in serum-free medium (300 µl containing 1×10^5^ cells) were added to the top chamber. The bottom chamber was prepared using 10% FBS, whichacted as a chemo-attractant. After 48 h of incubation, the non-migrative cells were removed with a cotton swab. Methanol was used to fix the cells that migrated through the membrane and stuck to the membrane's lower surface.After fixing the cells with methanol, haematoxylin was used for the purpose of staining. For quantification, the cells were counted under a microscope in five predetermined fields at ×200.

### Tumour cell invasion assay

Invasion assays were performed using the cell invasion chamber (BD, USA) according to the manufacturer's protocol. In this case, warm serum-free medium was added to the top of the cell invasion chamber. The serum-free medium rehydrated the ECM layer for 2 h at room temperature. Tumor cells in serum-free medium (300 µl containing 1×10^5^ cells) were added to the top chamber. The bottom chamber was prepared using 10% FBS, whichacted as a chemo-attractant. After 48 h of incubation, the non-invasive cells were removed with a cotton swab. Methanol was used to fix the cells that migrated through the membrane and stuck to the membrane's lower surface.After fixing the cells with methanol, haematoxylin was used for the purpose of staining. For quantification, the cells were counted under a microscope in five predetermined fields at ×200.

### Statistical analysis

Fisher's exact test was used to evaluate the correlation of HMGB1 expression with various clinicopathological parameters. Overall survival was calculated from the date of surgery to the date of death. Kaplan-Meier method was used to perform survival analyses. Cox proportional-hazard analysis was used for performing univariate and multivariate analysis: these kinds of analysis were used to explore the effect of variables on survival. SPSS 13.0 software was used for performing all kinds of statistical analyses.In this study, a *p* value of <0.05 was considered significant.

## Results

The evaluated and determined standard of curativity is those persons whose survival over five-year. According to our analysis, the curativity is 43/208 (20.67%).

### HMGB1 is overexpressed in HCC tissues

HMGB1 expression was determined by IHC in the 208 surgical specimens of HCC. An overexpression of HMGB1 was exhibited in 134 (64.4%) surgical specimens, whereas downexpression of HMGB1 was reported in the remaining 74 cases (35.6%, Table 1). As shown in Figure 1, the immunoreactivity of HMGB1 was detected at variable levels and localized within the cellular nuclei and cytoplasm. The HMGB1 protein expression was negative in normal liver tissues. On the other hand, HMGB1 protein expression was weak in cirrhotic liver, while strong expression of HMGB1 protein was detected in HCC tissues (Fig. 1). However, the statistical evaluation of immunohistochemical checking revealed that there was no statistically significant relationship between HMGB1 expression and clinicopathological parameters derived from clinical materials, follow-up data, and pathological findings.

**Figure 1:** Expressions of HMGB1 in HCC tissues and surrounding non-cancerous tissues. (A) Negative expression in distant normal liver tissue (IHC ×200). (B) Weak expression in HCC tissues (IHC ×400). (C) Moderate expression in HCC tissues (IHC ×400). (D) Strong expression in HCC tissues (IHC ×400). (E) Weak expression in cirrhotic liver (IHC ×200). (F) HCC tissue (HE ×200).

**Table 1:** Relationship between hmgb1 expression and clinicopathologic features of hcc patients.

Features	n	HMGB1	Expression	*p* value
		High	Low	
All cases	208	134	74	
Age(years)				0.386
<50	115	71	44	
≥50	93	63	30	
Gender				0.839
Male	178	114	64	
Female	30	20	10	
Tumor size(cm)				0.747
<5	57	38	19	
≥5	151	96	55	
Tumor number				0.119
single	142	86	56	
multiple	66	48	18	
Liver cirrhosis				0.468
Yes	65	46	19	
No	82	51	31	
Metastasis				0.619
Yes	53	36	17	
No	155	98	57	
Recurrence				0.767
Yes	81	51	30	
No	127	83	44	
HBsAg status				0.839
Positive	177	113	64	
Negative	31	21	10	
Serum AFP (ng/ml)				0.041*
<400	114	66	48	
≥400	94	68	26	
CLIP				0.007*
0	16	7	9	
1	33	15	18	
2	57	35	22	
3	53	39	14	
4	49	38	11	

*Statistically significant (p<0.05). The Fisher's exact test was used for comparison between groups.

### Correlation between HMGB1 expression and patients' survival

While differentiating patients with high and low HMGB1 protein levels, we correlated the prognostic effect of HMGB1 withthe overall survival of HCCpatients. By Kaplan-Meier curve assessment, it was found that high HMGB1 protein level was a significant prognostic factor in deciphering the poor overall survival in HCC patients. Patients with high HMGB1 protein level had a significantly lower 5-year survival rate than those with low HMGB1 protein level (Fig. 2, *p*<0.05). While comparing the Kaplan-Meier survival curves for low IHC expressions and high IHC expressions of HMGB1, we found a significant separation (*p* = 0.001, log-rank test) in the 208 HCC patients.

**Figure 2:** Kaplan-Meier survival analysis of primary HCC patients (n = 208) after surgical resection with high HMGB1 expression (n = 134) and low HMGB1 expression (n = 74). The survival rate for patients in the HMGB1-high group was significantly lower than that for patients in the HMGB1-low group (log-rank, *p* = 0.001).

### Univariate and multivariate analyses of prognostic variables in HCC patients

To identify the variables with potential prognostic significance, univariateanalysis of each variable was performed in relation to the survival time of patients with HCC. The difference in predicting the prognosis was assessed by examining the ratio hazard and *p* value for each variable. Then, the relative importance of each variable was determined by multivariate Cox proportional hazards model analysis. The stepwise inclusion of variables in the model was performed through univariate analysis, which proved that the significant prognostic factors were HMGB1 expression, gender, tumor size, tumor number, CLIP and serum AFP in the over survival (OS) and time to recurrence (TTR) of HCC patients. Multivariate analysis results showed that the OS of HCC patients could be predicted on the basis of significant prognostic factors, such as HMGB1 expression, gender, tumor size, tumor number, CLIP and serum AFP (Table 2). Multivariate analysis results showed that the TTR of HCC patients could be predicted on the basis of significant prognostic factors, such as HMGB1, gender, CLIP and tumor number. (Table 3).

**Table 2:** Univariate and multivariate analyses of individual parameters for correlations with os rate: cox proportional hazards model.

Variables	Univariable			Multivariable		
	HR	CI (95%)	*p* value	HR	CI (95%)	*p* value
HMGB1	0.568	0.398–0.811	0.002*	0.562	0.388–0.815	0.002*
Age(years)(<50 vs. ≥50)	1.074	0.772–1.495	0.672			
Gender	0.410	0.232–0.726	0.002*	0.539	0.302–0.963	0.037*
Tumor Size(cm)(<5 vs. ≥5)	0.636	0.433–0.934	0.021*			
Tumor number(single vs multiple)	0.045	0.028–0.071	<0.001*	0.060	0.036–0.101	<0.001*
Liver cirrhosis	1.259	0.836–1.895	0.271			
AFP(ng/ml)(<400 vs. ≥400)	0.512	0.369–0.711	<0.001*			
CLIP	1.900	1.621–2.228	<0.001*	1.330	1.117–1.582	0.001*

Abbreviations: HR, Hazard radio; CI, Confidence interval. os, overall survival.

*Statistically significant (p<0.05).

**Table 3:** Univariate and multivariate analyses of individual parameters for correlations with ttr rate: cox proportional hazards model.

Variables	Univariable			Multivariable		
	HR	CI (95%)	*p* value	HR	CI (95%)	*p* value
HMGB1	0.574	0.402–0.820	0.002*	0.611	0.422–0.884	0.009*
Age(years)(<50 vs. ≥50)	1.004	0.990–1.017	0.587			
Gender	0.409	0.231–0.725	0.002*	0.518	0.290–0.925	0.026*
Tumor Size(cm)(<5 vs. ≥5)	0.633	0.431–0.930	0.020*			
Tumor number(single vs multiple)	0.052	0.033–0.081	<0.001*	0.072	0.044–0.120	<0.001*
Liver cirrhosis	1.060	0.764–1.469	0.728			
AFP(ng/ml)(<400 vs. ≥400)	0.519	0.374–0.720	<0.001*			
CLIP	1.912	1.630–2.242	<0.001*	1.363	1.145–1.622	<0.001*

Abbreviations: HR, Hazard radio; CI, Confidence interval. ttr, time to recurrence.

*Statistically significant (p<0.05).

### Expression of HMGB1 in HCC cells by real-time PCR and Western blot

Real-time PCR and Western blot techniques were performed in the human HCC cell lines HepG2, M6, Huh7, 97H, 97L, M3, BEL-7404, and a normal hepatocyte line (L02). Compared with the normal heptocyte line, all the 6 HCC cell lines showed higher level expression of HMGB1 mRNA (Fig. 3A). Furthermore, western blot technique revealed that HMGB1 was overexpressed in most HCC cell lines. In contrast, HMGB1 expression was undetectable in the normal hepatocyte line (Fig. 3B).

**Figure 3:** Expression analysis of HMGB1 mRNA and protein in normal hepatocyte line (L02) and HCC cell lines (HCCLM3, Huh7, HepG2, HCCLM6, MHCC97H, MHCC97L, BEL-7404) by real-time PCR (A) and Western blotting (B).

### HMGB1 expression in interfered HCC cells by real-time PCR and Western blot

To further determine whether HMGB1 expression plays a role in human HCC cell invasion, an RNA interference technique was used to knock down endogenous HMGB1. After introducing HMGB1 siRNA into M6 cell, it was found that HMGB1 expression reduced within 48 h after transfection.Moreover, non-specific siRNA did not substantially affect the expression of endogenous HMGB1 (Fig. 4A and B).

**Figure 4:** HMGB1 expression in interfered HCC cells. (A)Western blot was performed to determine HMGB1 protein expression in HCCLM6, HCCLM6/mock, HCCLM6/S1, HCCLM6/S2, HCCLM3,HCCLM3/mock,HCCLM3/HMGB1^+^); Tubulin was used as a control. (B)qRT-PCR was performed to determined HMGB1 mRNA expresion in HCCLM6, HCCLM6/mock, HCCLM6/S2, HCCLM3, HCCLM3/mock, HCCLM3/HMGB1^+^).

On the other hand, plasmid human HMGB1 DNA was used to enhance endogenous HMGB1 expression. After introducing the HMGB1 DNA into M3 cell, we found that HMGB1 expression enhanced within 48 h after transfection.Moreover,the vector GV142 did not substantially affect the expression of endogenous HMGB1 (Fig. 4A and B).

### Alteration of HMGB1 expression regulated proliferation, migration and invasion capabilities of HCC cells

Compared to HMGB1 siRNA S1, HMGB1 siRNA S2 was more effective in silencing HMGB1 protein. Therefore, we used HMGB1 siRNA S2 to perform our experiments. Compared with its controls (M6 and M6/mock), M6/S2, HMGB1 knockdown cells exhibited significantly lower proliferation, migration and invasion tendencies during these cell assays (*p*<0.05; Fig. 5, 6 and 7).

**Figure 5:** Effect of HMGB1 on cell growth. CCK-8 assay showed that inhibition of HMGB1 expression in HCCLM6 cells significantly reduced cell viability, while overexpression of HMGB1 in HCCLM3 cells accelerated cells viability.

**Figure 6:** Cell migration assay. The number of cells that passed through cell chamber in HCCLM6/S2 group was less than in two other groups. However, the number of cells that passed through cell chamber in HCCLM3/HMGB1^+^ group was more than in two other groups. All the results were represented as the mean ± SD from three independent experiments. *p<0.05 (compared with both parental and mock groups). Migrating cells were stained with Giemsa and visualized by microscopy (original magnification ×200).

**Figure 7:** Cell invation assay. The number of cells that passed through Matrigel in HCCLM6/S2 group was less than in two other groups. However, the number of cells that passed through Matrigel in HCCLM3/HMGB1^+^ group was more than in two other groups. All the results were represented as the mean ± SD from three independent experiments. *p<0.05 (compared with both parental and mock groups). Invating cells were stained with Giemsa and visualized by microscopy (original magnification ×200).

On the other hand, plasmid human HMGB1 DNA was used to enhance endogenous HMGB1 expression. Compared with its controls (M3 and M3/mock), the enhancement of HMGB1 expression in cells exhibited significantly enhanced proliferation, migration and invasion tendencies during these cell assays (*P*<0.05; Fig. 5, 6 and 7).

## Discussion

There have been major breakthroughs in the diagnosis and chemotherapy measures used in the treatment of cancer. However, HCC continues to be one of the most deadly human carcinomas, and the prognosis of HCC remains dismal [28].In clinical practice, prognostic molecular biomarkers are valuable toolsin predicting the progression of disease in patients. And these patients we selected are at early or intermediate stage of hepatocellular carcinoma patients in our study. Clinicians use these prognostic biomarkers in planning strategies that control the proliferation of tumor.

In this study, we determined the HMGB1 expression in HCC patients. We also explored the clinical prognostic significance of HMGB1 expression. For this purpose, we analyzed the entire long-term follow-up data of a large cohort of HCC patients along with their corresponding clinical samples. We have found that the HMGB1 protein is expressed much more strongly in almost all HCCs than in normal liver and cirrhotic liver tissues. We also found the overexpression of HMGB1 protein at the transcriptional and translational levels of HCC cell lines. Our results also indicate that HMGB1 probably plays a role in hepatocarcinogenesis.However,we could not completely elucidate the precise molecular mechanism of HMGB1 in HCC tumorigenesis. The findings of HMGB1 overexpression in our study are in good agreement with most observations reported in previous cancer studies. In summary, our study confirms a close association of HMGB1 expression with the genesis and development of tumors.

Several research studies have reported that HMGB1 plays a pivotal role in cancer progression. Kuniyasu *et al* [29] reported that HMGB1 was highly expressed in gastric cancer and that its receptor, RAGE, was closely associated with the invasion and metastasis of gastric cancer. Volp *et al* [24] reported that significantly elevated levels of HMGB1 expression were found in colon carcinoma compared with that detected in corresponding normal tissues. Using the colitis-associated cancer model, Maeda *et al* [30] showed that the incidence and growth of tumor could be decreased by neutralizing anti-HMGB1 antibody, which inhibited the expression of HMGB1.Our contingency table analysis, however, showed that HMGB1 expression does not correlate with any of the clinicopathological parameters analyzed in this study, but AFP. On the other hand, our Kaplan-Meier survival analysis revealed that high level HMGB1 expression was significantly linked with a poor prognosis of HCC patients after surgical resection.When the expression of HMGB1 was higher, the survival time for HCC patients was found to be shorter. The univariate analysis of Cox proportional-hazard model proved that significant prognostic factors, such as HMGB1 expression, tumor size, recurrence, metastasis, and serum AFP were associated with an increased risk of death from HCC. In contrast, multivariate analysis proved that HMGB1 expression, gender, tumor size, recurrence, metastasis, and serum AFPwere thesix significant and independent prognostic factors that could be associated with overall survival of HCC patients. Barring HMGB1 expression, the other factors are well-acknowledged indicators of HCC. As HMGB1 expression is now considered as anovel and independent predictor of decreased disease-free survival of patients with prostate cancer, it may also be reckoned as a new and independent predictor of prognosis for HCC patients.

Metastasis is regarded as the main cause of death in cancer patients [31]. For HCC patients, the intrahepatic and distant metastasis has been considered as the primary factor for poor prognosis. The metastatic process includes a series of interdependent events, including cancer cell proliferation, migration, and invasion [32]. As a nuclear protein, HMGB1 plays the dual roles of being a chromatin structural protein and a cytokine [33], [34]. It is involved in various processes of cancer progression, including cell proliferation, angiogenesis, invasion, and metastasis [35]. In this study, we proved that the down-regulation of HMGB1 inhibits the invasion of HCCLM6 cells, whereas the up-regulation of HMGB1 enhances the invasion of HCCLM3 cells.

In summary, our study evaluated the prognostic significance of HMGB1 expression in numerousspecimens of HCC clinical tissues. As these patients we selected are at early or intermediate stage of HCC patients in our study, the prognostic significance of HMGB1 is related with a part of HCC patients. Immunohistochemical analysis was used to evaluate HMBG1 expression at protein level in these HCC clinical samples. We detected the overexpression of HMGB1 in both HCC cell lines and HCC tissues: the overexpression of HMGB1 was found at both the transcriptional and translational levels. Moreover, the overall survival of our study cohort was significantly poorer in high HMGB1 expression cases than in low HMGB1 expression cases. Therefore, we can infer that HMGB1 expression is a new and independent predictor for HCC patients. Our results indicate that the down-regulation of HMGB1 inhibits the proliferation, migration and invasion of HCCLM6 cells, whereas the up-regulation of HMGB1 enhances the proliferation, migration and invasion of HCCLM3 cells. Our finding also provides evidence for molecular target therapy of tumor. In order to completely elucidate the mechanism of carcinogenesis and tumor progression in patients with HCC, further molecular, cellular, and animal model studies should be conducted.

## References

[1] LlovetJM, BurroughsA, BruixJ (2003) Hepatocellular carcinoma. Lancet 362: 1907–17.1466775010.1016/S0140-6736(03)14964-1

[2] BlockTM, MehtaAS, FimmelCJ, JordanR (2003) Molecular viral oncology of hepatocellular carcinoma. Oncogene 22: 5093–107.1291024710.1038/sj.onc.1206557

[3] Tung-Ping PoonR, FanST, WongJ (2000) Risk factors, prevention, and management of postoperative recurrence after resection of hepatocellular carcinoma. Ann Surg 232: 10–24.1086219010.1097/00000658-200007000-00003PMC1421103

[4] CapocacciaR, SantM, BerrinoF, SimonettiA, SantiV, et al (2007) Hepatocellular carcinoma: trends of incidence and survival in Europe and the United States at the end of the 20th century. Am J Gastroenterol 102: 1661–70 quiz 0, 71.1755545910.1111/j.1572-0241.2007.01337.x

[5] El-SeragHB (2004) Hepatocellular carcinoma: recent trends in the United States. Gastroenterology 127: S27–34.1550809410.1053/j.gastro.2004.09.013

[6] ThomasMB, ZhuAX (2005) Hepatocellular carcinoma: the need for progress. J ClinOncol 23: 2892–9.10.1200/JCO.2005.03.19615860847

[7] LoCM, NganH, TsoWK, LiuCL, LamCM, PoonRT, et al (2002) Randomized controlled trial of transarteriallipiodol chemoembolization for unresectable hepatocellular carcinoma. Hepatology 35: 1164–71.1198176610.1053/jhep.2002.33156

[8] NgKK, LoCM, LiuCL, PoonRT, ChanSC, et al (2008) Survival analysis of patients with transplantable recurrent hepatocellular carcinoma: implications for salvage liver transplant. Arch Surg 143: 68–74 1820915510.1001/archsurg.2007.15

[9] Kim doY, PaikYH, AhnSH, YounYJ, ChoiJW, et al (2007) PIVKA-II is a useful tumor marker for recurrent hepatocellular carcinoma after surgical resection. Oncology (Suppl 1) 52–7.10.1159/00011170718087182

[10] UlloaL (2005) The vagus nerve and the nicotinic anti-inflammatory pathway. Nat Rev Drug Discov 4: 673–84.1605639210.1038/nrd1797

[11] UlloaL, TraceyKJ (2005) The “cytokine profile”: a code for sepsis. Trends Mol Med 11: 56–63.1569486710.1016/j.molmed.2004.12.007

[12] LotzeMT, TraceyKJ (2005) High-mobility group box 1 protein (HMGB1): nuclear weapon in the immune arsenal. Nat Rev Immunol 5: 331–42.1580315210.1038/nri1594

[13] UlloaL, BatliwallaFM, AnderssonU, GregersenPK, TraceyKJ (2003) High mobility group box chromosomal protein 1 as a nuclear protein, cytokine, and potential therapeutic target in arthritis. Arthritis Rheum 48: 876–81.1268752810.1002/art.10854

[14] MullerS, RonfaniL, BianchiME (2004) Regulated expression and subcellular localization of HMGB1, a chromatin protein with a cytokine function. J Intern Med 255: 332–43.1487145710.1111/j.1365-2796.2003.01296.x

[15] BianchiME (2004) Significant (re)location: how to use chromatin and/or abundant proteins as messages of life and death. Trends Cell Biol 14: 287–93.1518318510.1016/j.tcb.2004.04.004

[16] UlloaLuis, MessmerDavorka (2006) High-mobility group box 1 (HMGB1) protein: Friend and foe. Cytokine & Growth Factor Reviews 17: 189–201.1651340910.1016/j.cytogfr.2006.01.003

[17] M.T. LotzeKJ (2005) Tracey, High-mobility group box 1 protein (HMGB1): nuclear weapon in the immune arsenal,. Nat Rev Immunol 5: 331–342.1580315210.1038/nri1594

[18] MullerS, ScaffidiP, DegryseB, BonaldiT, RonfaniL, et al (2001) Bianchi, New EMBO members' review: the double life of HMGB1 chromatin protein: architectural factor and extracellular signal. EMBO J 20: 4337–4340.1150036010.1093/emboj/20.16.4337PMC125571

[19] DongXD, ItoN, LotzeMT, DemarcoRA, PopovicP, et al (2007) High mobility group box 1(HMGB1) release from tumor cells after treatment: implications for development of targeted chemoimmunotherapy. Immunother 30: 596–606.10.1097/CJI.0b013e31804efc7617667523

[20] EllermanJE, BrownCK, de VeraM, ZehHJ, BilliarT, et al (2007) Masquerader: high mobility group box-1 and cancer, Clin. Cancer Res 13: 2836–2848.10.1158/1078-0432.CCR-06-195317504981

[21] BrezniceanuML, VolpK, BosserS, SolbachC, LichterP, et al (2003) HMGB1 inhibits cell death in yeast and mammalian cells and is abundantly expressed in human breast carcinoma. FASEB J 17: 1295–1297.1275933310.1096/fj.02-0621fje

[22] PoserI, GolobM, BuettnerR, BosserhoffAK (2003) Upregulation of HMG1 leads to melanoma inhibitory activity expression in malignant melanoma cells and contributes to their malignancy phenotype. Mol Cell Biol 23: 2991–2998.1266559510.1128/MCB.23.8.2991-2998.2003PMC152547

[23] AkaikeH, KonoK, SugaiH, TakahashiA, MimuraK, et al (2007) Expression of high mobility group box chromosomal protein-1 (HMGB-1) in gastric cancer. Anticancer Res 27: 449–457.17352266

[24] VolpK, BrezniceanuML, BosserS, BrabletzT, KirchnerT, et al (2006) Increased expression of high mobility group box 1 (HMGB1) is associated with an elevated level of the antiapoptotic c-IAP2 protein in human colon carcinomas. Gut 55: 234–242.1611835210.1136/gut.2004.062729PMC1856519

[25] ChoiYR, KimH, KangHJ, KimNG, KimJJ, et al (2003) Overexpression of high mobility group box 1 in gastrointestinal stromal tumors with KIT mutation. Cancer Res 63: 2188–2193.12727838

[26] YongfengXu, YongYi, ShuangjianQiu (2010) PEBP1 downregulation is associated to poor prognosis in HCC related to hepatitis B infection. Journal of Hepatology 53: 872–879.2073908310.1016/j.jhep.2010.05.019

[27] WuD, DingY, WangS, ZhangQ, LiuL (2008) Increased expression of high mobility group box 1(HMGB1) is associated with progression and poor prognosis in human nasopharyngeal carcinoma. J Pathol 216: 167–175.1868013710.1002/path.2391

[28] ZhangHK, PanK, WangH, WengDS, SongHF, et al (2008) Decreased expression of ING2 gene and its clinicopathological significance in hepatocellular carcinoma. Cancer Lett 261: 183–192.1816021210.1016/j.canlet.2007.11.019

[29] KuniyasuH, OueN, WakikawaA, ShigeishiH, MatsutaniN, et al (2002) Expression of receptors for advanced glycation end-products (RAGE) is closely associated with the invasive and metastatic activity of gastric cancer. J Pathol 196: 163–170.1179336710.1002/path.1031

[30] MaedaS, HikibaY, ShibataW, OhmaeT, YanaiA, et al (2007) Essential roles of high-mobility group box 1 in the development of murine colitis and colitis-associated cancer. BiochemBiophys Res Commun 360: 394–400.10.1016/j.bbrc.2007.06.06517599806

[31] RudmikLR, MaglioccoAM (2005) Molecular mechanisms of hepatic metastasis in colorectal cancer. J SurgOncol 92: 347–359.10.1002/jso.2039316299807

[32] KumarS, WeaverVM (2009) Mechanics, malignancy, and metastasis: the force journey of a tumor cell. Cancer Metastasis Rev 28: 113–127.1915367310.1007/s10555-008-9173-4PMC2658728

[33] NaghaviMH, NowakP, AnderssonJ (2003) Intracellular high mobility group B1 protein(HMGB1) represses HIV-1 LTRdirected transcription in a promoter- and cell-specific manner. Virology 314: 179–189.1451707110.1016/s0042-6822(03)00453-7

[34] KostovaN, ZlatevaS, UgrinovaI, PashevaE (2010) The expression of HMGB1 protein and its receptor RAGE in human malignant tumors. Mol Cell Biochem337: 251–258.10.1007/s11010-009-0305-019876719

[35] TangD, KangR, ZehHJ, LotzeMT (2010) High-mobility group box 1 and cancer. BiochimBiophysActa 1799: 131–140.10.1016/j.bbagrm.2009.11.014PMC281855220123075

